# Identification of Prognostic Fatty Acid Metabolism lncRNAs and Potential Molecular Targeting Drugs in Uveal Melanoma

**DOI:** 10.1155/2022/3726351

**Published:** 2022-10-11

**Authors:** Yang Xu, Rui Tian, Xin Liu, Meijiao Song, Lu Liu, Rong Guo, Zhuoya Li, Xiaomin Hu, Hui Zhang

**Affiliations:** ^1^Jilin University, Hospital Stomatol, Jilin Provincial Key Laboratory Tooth Development & Bone Remodeling, 763 Heguang Rd., Changchun, 130021 Jilin Province, China; ^2^Department of Ophthalmology, The Second Hospital of Jilin University, Changchun, 130041 Jilin Province, China

## Abstract

**Background:**

The aim of this study was to identify prognostic fatty acid metabolism lncRNAs and potential molecular targeting drugs in uveal melanoma through integrated bioinformatics analysis.

**Methods:**

In the present study, we obtained the expression matrix of 309 FAM-mRNAs and identified 225 FAM-lncRNAs by coexpression network analysis. We then performed univariate Cox analysis, LASSO regression analysis, and cross-validation and finally obtained an optimized UVM prognosis prediction model composed of four PFAM-lncRNAs (AC104129.1, SOS1-IT1, IDI2-AS1, and DLGAP1-AS2).

**Results:**

The survival curves showed that the survival time of UVM patients in the high-risk group was significantly lower than that in the low-risk group in the train cohort, test cohort, and all patients in the prognostic prediction model (*P* < 0.05). We further performed risk prognostic assessment, and the results showed that the risk scores of the high-risk group in the train cohort, test cohort, and all patients were significantly higher than those of the low-risk group (*P* < 0.05), patient survival decreased and the number of deaths increased with increasing risk scores, and AC104129.1, SOS1-IT1, and DLGAP1-AS2 were high-risk PFAM-lncRNAs, while IDI2-AS1 were low-risk PFAM-lncRNAs. Afterwards, we further verified the accuracy and the prognostic value of our model in predicting prognosis by PCA analysis and ROC curves.

**Conclusion:**

We identified 24 potential molecularly targeted drugs with significant sensitivity differences between high- and low-risk UVM patients, of which 13 may be potential targeted drugs for high-risk patients. Our findings have important implications for early prediction and early clinical intervention in high-risk UVM patients.

## 1. Introduction

Uveal melanoma (UVM) is the most common intraocular malignant tumor, accounting for the first place of intraocular tumors [1]. This tumor is more common in adults, with a high degree of malignancy. The posterior pole of the eye is a predilection site, easy to transfer through blood flow, and the prognosis is poor [2, 3]. The occurrence and development of UVM is a complex process involving multifactor, multistage, and multigene variation accumulation and interaction [4]. It is widely believed that the abnormal expression of oncogenes and tumor suppressor genes leads to malignant transformation of cells, and these genes usually play a key role in the regulation of cell proliferation, division, and differentiation [5].

Metabolic dysregulation is one of the ten hallmarks of cancer, and increasing evidence suggests that metabolic reprogramming plays a crucial role in cancer initiation and progression [6, 7]. As an important part of lipid metabolism, fatty acids can accumulate to meet the needs of lipid synthesis signaling molecules and membranes [8]. Unregulated fatty acids can not only interfere with the efficacy of chemotherapy and radiotherapy in cancer patients but also affect immunotherapy, which is a breakthrough in tumor therapy in recent years [9, 10].

More and more studies have shown that fat metabolism has a certain relationship with the occurrence and development of tumors, and fatty acid metabolism (FAM) is crucial for the maintenance of the malignant tumor microenvironment [11–13]. In this paper, the correlation between fatty acid metabolism genes (FAMGs) and UVM was discussed, a prognosis prediction model based on FAMGs was constructed, and molecular targeted drugs sensitive to high-risk UVM patients were screened. Our findings have important implications for early prediction and early clinical intervention in high-risk UVM patients.

## 2. Materials and Methods

### 2.1. Data Download and Collation

Transcriptome data of UVM and corresponding clinical data were downloaded from our TCGA database (https://tcga-data.nci.nih.gov/tcga) [14], and a total of 80 UVM samples were collected. We then used custom Perl scripts to clean up all the data for subsequent analysis.

### 2.2. Identification of Fatty Acid Metabolism lncRNAs by Coexpression Analysis

First, the transcriptome expression matrices of all UVM samples were classified as RNAs, and mRNA and lncRNA expression matrices were screened out. Then, the relative expression levels of fatty acid metabolism genes (FAMGs) were extracted from the UVM transcriptome gene matrix using the R package limma [15]. Finally, the coexpression analysis of fatty acid metabolism mRNAs (FAM-mRNAs) and lncRNAs (FAM-lncRNAs) was performed by Pearson correlation test to determine the FAM-lncRNAs [16]. Pearson correlation coefficient > 0.7 and *P* value < 0.01 were considered statistically significant.

### 2.3. Construction of UVM Prognostic Prediction Model

First, the expression matrix of FAM-lncRNAs was collated and combined with the survival time and survival status of UVM patients. Then, all samples were randomly divided into the train cohort and the test cohort. Univariate and multivariate analyses and LASSO regression analysis were used to construct the UVM prognostic prediction model [17]. The relative expression levels of FAM-lncRNAs in each sample were then multiplied by the risk factors and added together to obtain the risk score for each sample [18]. Finally, by comparing the risk score of each sample with the median risk score of the model, all patients can be divided into the high-risk group and the low-risk group [19].

### 2.4. Survival Analysis of UVM Patients with Different Risk Groups

We performed a survival analysis of patients in the high-risk and low-risk groups to explore the prognostic value of prognostic prediction models [20]. We organized the train cohort, test cohort, and all patients' survival information, risk score, risk grouping, and FAM-lncRNA expression matrix and plotted the survival curve of UVM patients in high- and low-risk groups to show the difference in survival prognosis of patients in different risk groups [21].

### 2.5. Risk Assessment of UVM Patients with Different Risk Groups

We performed risk assessments of UVM patients in high- and low-risk groups, aiming to elucidate the correlation between patient survival time, survival status, FAM-lncRNA expression, and risk score. Results are presented as risk curves, survival scatter plots, and risk gene heat maps [22, 23].

### 2.6. Principal Component Analysis of UVM Patients with Different Risk Groups

To further verify whether our model can accurately distinguish between high-risk and low-risk UVM patients, we performed a principal component analysis (PCA) [24]. PCA is a statistical method that converts a group of possibly correlated variables into a group of linearly unrelated variables through orthogonal transformation [25]. The transformed variables are called principal components. We performed PCA of FAMGs and model genes by R package limma and ggplot2, respectively, and visualized them with scatter plots [26, 27].

### 2.7. ROC Curve Analysis of UVM Prognosis Prediction Model

Receiver Operating Characteristic (ROC), also known as the sensitivity curve, is a comprehensive index reflecting the continuous variables of sensitivity and specificity, and the relationship between the two is usually represented by a curve graph [28, 29]. The area under the ROC curve (AUC) represents the accuracy of a diagnostic test [30]. We used the R packages survival, survminer, and timeROC to test the accuracy of the UVM prognostic prediction model and plotted the ROC curves of the survival rate and clinical characteristics for visualization [31, 32].

### 2.8. Screening of Potential Molecular Targeting Drugs for UVM

In order to screen potential molecular targeting drugs for UVM, sensitivity analysis was performed on the whole transcription gene expression matrix and drugs through R package limma, ggpubr, pRRopetic, and ggplot2, and then, the UVM risk file and drug sensitivity results were combined to compare the sensitivity differences of patients in the high- and low-risk groups to different drugs [33]. Finally, we visualize the results through a boxplot. Finally, potential molecular targeted drugs for UVM were screened by drug sensitivity analysis [34].

## 3. Results

### 3.1. Identification of FAM-lncRNAs

We downloaded and collated 60,660 RNA transcript expression matrices from the TCGA database, including 19,962 mRNAs and 16,901 lncRNAs. We then obtained the expression matrix of 309 FAM-mRNAs and identified 225 FAM-lncRNAs by coexpression network analysis. The expression matrix of FAM-lncRNAs and their coexpression relationship with FAM-mRNAs are shown in Supplementary File 1.

### 3.2. Prognostic Prediction Model for UVM Patients

Univariate Cox analysis was performed on 225 FAM-lncRNAs, and 25 prognosis-related FAM-lncRNAs (PFAM-lncRNAs) were obtained, of which 4 PFAM-lncRNAs were low-risk lncRNAs (hazard ratio < 1) and 21 were high-risk lncRNAs (hazard ratio > 1) (as shown in Figure 1(a)). LASSO regression was used to select five PFAM-lncRNAs with significant differential expression to construct a Cox prognostic model (Figures 1(b) and 1(c)). The prognosis prediction model was evaluated and optimized by cross-validation, and finally, an optimized model consisting of four PFAM-lncRNAs (AC104129.1, SOS1-IT1, IDI2-AS1, and DLGAP1-AS2) was obtained. The raw data related to the prognostic prediction model are detailed in Supplementary File 2.

### 3.3. Differences in Survival Prognosis of Patients with Different UVM Risk Groups

Survival curves were drawn by comparing the survival differences between the high-risk and low-risk groups in the train cohort, test cohort, and all patients in the prognostic prediction model. As shown in Figures 2(a)–2(c), the survival time of UVM patients in the high-risk group was significantly lower than that in the low-risk group (*P* < 0.05).

### 3.4. Differences in Risk Prognosis of Patients with Different UVM Risk Groups

We further performed risk prognostic assessment to predict the risk prognostic of UVM patients in the high-risk and low-risk groups. The risk scores of the high-risk group in the train cohort, test cohort, and all patients were significantly higher than those of the low-risk group (*P* < 0.05) (Figures 3(a)–3(c)). As the risk score increased, patient survival decreased and the number of deaths increased (Figures 3(d)–3(f)). As shown in Figures 3(g)–3(i), AC104129.1, SOS1-IT1, and DLGAP1-AS2 were high-risk PFAM-lncRNAs, while IDI2-AS1 were low-risk PFAM-lncRNAs. These results suggest that the prognostic prediction model can accurately assess the difference in risk prognosis between patients in high- and low-risk groups.

### 3.5. PCA Analysis of the Prognostic Prediction Model

Through PCA analysis, we further verified the accuracy of our model in predicting prognosis. As shown in Figures 4(a) and 4(b), FAMGs and genes involved in model construction are highly discriminative between the high-risk group and low-risk group UVM patients, which indicates that the prognostic prediction model we constructed can better distinguish high-risk and low-risk patients.

### 3.6. ROC Curves of UVM Prognosis Prediction Model

We plotted ROC curves to assess and validate the prognostic value of the model. As shown in Figure 5(a), the AUCs for the 1-, 3-, and 5-year survival rates were 0.951, 0.953, and 1.000, respectively. Compared with other clinical features, the risk score AUC value based on the prognostic prediction model was the highest (1.000) (see Figure 5(b)). The above results demonstrate that the prognostic model can accurately and independently predict the prognosis of UVM patients.

### 3.7. Potential Molecular Targeted Drugs of UVM

Through drug sensitivity analysis, we identified 24 potential molecularly targeted drugs with significant sensitivity differences between high- and low-risk UVM patients (see Supplementary File 3 for details) (*P* < 0.05).  Figure 6 shows 13 molecularly targeted drugs, which have lower IC50 values in high-risk patients, indicating that these drugs may be potential molecularly targeted drugs for high-risk patients.

## 4. Discussion

UVM is the most common primary intraocular malignancy in adults, accounting for 85% of all ocular melanomas, and more than 50% of patients with UVM develop systemic metastases, which are rarely managed by surgery [35, 36]. The curative effect of UVM therefore often leads to a poor prognosis [37]. In this paper, we obtained the expression matrix of 309 FAM-mRNAs and identified 225 FAM-lncRNAs by coexpression network analysis. We then performed univariate Cox analysis, LASSO regression analysis, and cross-validation and finally obtained an optimized UVM prognosis prediction model composed of four PFAM-lncRNAs (AC104129.1, SOS1-IT1, IDI2-AS1, and DLGAP1-AS2). Next, we drew survival curves, showing that the survival time of UVM patients in the high-risk group was significantly lower than that in the low-risk group in the train cohort, test cohort, and all patients in the prognostic prediction model (*P* < 0.05). We further performed risk prognostic assessment, and the results showed that the risk scores of the high-risk group in the train cohort, test cohort, and all patients were significantly higher than those of the low-risk group (*P* < 0.05), patient survival decreased and the number of deaths increased with increasing risk scores, and AC104129.1, SOS1-IT1, and DLGAP1-AS2 were high-risk PFAM-lncRNAs, while IDI2-AS1 were low-risk PFAM-lncRNAs. Afterwards, we further verified the accuracy and the prognostic value of our model in predicting prognosis by PCA analysis and ROC curves. Finally, we identified 24 potential molecularly targeted drugs with significant sensitivity differences between high- and low-risk UVM patients, of which 13 may be potential targeted drugs for high-risk patients.

To the best of our knowledge, there are no bioinformatics studies on the association of FAMGs with UVM. However, in recent years, studies have found that FAM is involved in the pathophysiological mechanism of UVM, thereby affecting the prognosis of patients. Han et al. [38] showed by RNA sequencing, metabolomics, and molecular analysis that oxidative phosphorylation of BRCA1-associated protein 1 (OXPHOS BAP1) mutant UVM cells utilizes glycolysis and nucleotide biosynthesis pathways and fatty acid oxidation pathways, while the loss of BAP1 live mutations is associated with the transfer of UVM. This suggests that targeting tumor metabolism is a potential therapeutic option for BAP1-mutant UVM. Gu et al. [39] found that oridonin inhibited the expression of fatty acid synthase (FAS) in UVM cells and enhanced the expression of FAS by insulin, partially rescued oridonin-induced apoptosis, and exhibited a strong anticancer effect. Using gas chromatography-mass spectrometry and spectrophotometry to compare the antioxidant status of uveal melanocytes and UVM cells, Blasi et al. [40] showed that the proportion of polyunsaturated fatty acids was significantly higher in UVM cells (*P* = 0.022), which showed that the antioxidant pattern of UVM cells is different from that of skin melanocytes, which may be one of the pathogenic mechanisms of abnormal proliferation of UVM cells.

Using comprehensive bioinformatics analyses, we identified FAM-lncRNAs by coexpression analysis, constructed a UVM prognostic prediction model, performed survival analysis and risk assessment of UVM patients with different risk groups, and further verified the accuracy and prognostic value of our model in predicting prognosis by PCA analysis and ROC curves. Finally, we screened potential molecular targeting drugs for UVM through drug sensitivity analysis. Our findings will help to identify new prognostic lncRNA characteristics of UVM and potential molecular targeting drugs, which may have substantial clinical value for the early detection and early treatment of UVM patients, especially high-risk patients. However, this study also has some limitations, such as not paying attention to the characteristics of different pathological subtypes and clinical staging and grading of UVM and lack of experimental verification in vitro and in vivo. In the future, these are subject to our further research.

## Figures and Tables

**Figure 1:** (a) A forest plot of univariate regression analysis of 25 PFAM-lncRNAs of UVM patients. Green square: low hazard ratio (HR) value; red square: high HR value; blue solid lines represent 95% confidence intervals. Obtaining four PFAM-lncRNAs using optimal lambda value by the LASSO screening process (b) and cross-validation (c).

**Figure 2:** The survival curves of high- (red) and low-risk (blue) UVM patients in the train cohort (a), test cohort (b), and all patients (c). Abscissa: survival time of patients; ordinate: survival probability. The lists below the curves show the number of patients who survive each year.

**Figure 3:** Risk curves for the train cohort (a), test cohort (b), and all patients (c). Horizontal axis: patient risk score from low to high; vertical axis: risk score. Red dots represent high-risk groups; blue dots represent low-risk groups. Risk scatter plots for the train cohort (d), test cohort (e), and all patients (f). Vertical coordinate: survival time. Red dots indicate that the patient is dead; blue dots indicate that the patient is alive. Heat maps of risk for four PFAM-lncRNAs in the train cohort (g), test cohort (h), and all patients (i). Red squares represent highly expressed lncRNAs; blue squares represent lowly expressed lncRNAs.

**Figure 4:** Scatter plots for principal component analysis-based FAMGs (a) and genes involved in model construction (b). PC1: principal component 1; PC2: principal component 2. The red dots represent high-risk patients, and the blue dots represent low-risk patients.

**Figure 5:** ROC curves of UVM prognosis prediction model. The different colored curves represent different survival times (1, 3, and 5 years) (a) or clinical characteristics (b). AUC: area under the ROC curve. Abscissa: 1 − specificity (false positive rate); ordinate: sensitivity (true positive rate).

**Figure 6:** Boxplots of molecularly targeted drug sensitivity. Panels (a–m) show the differences in the sensitivity of different drugs in UVM patients with high- and low-risk groups. Red boxes represent the high-risk group; blue boxes represent the low-risk group. The abscissa indicates the grouping, and the ordinate indicates the drug sensitivity.

## Data Availability

The dataset used and/or analyzed during this study may be granted by contacting the corresponding author.

## Supplementary Materials

Supplementary Materials The expression matrix of FAM-lncRNAs and their coexpression relationship with FAM-mRNAs are shown in Supplementary File 1. The raw data related to the prognostic prediction model are detailed in the Supplementary File 2. Through drug sensitivity analysis, we identified 24 potential molecularly targeted drugs with significant sensitivity differences between high- and low-risk UVM patients (see Supplementary File 3 for details) (*P* < 0.05).
